# Targeted Diagnosis, Therapeutic Monitoring, and Assessment of Atherosclerosis Based on Mesoporous Silica Nanoparticles Coated with cRGD-Platelets

**DOI:** 10.1155/2022/6006601

**Published:** 2022-09-29

**Authors:** Wei Zhang, Zheng Lv, Yupeng Zhang, Subash C. B. Gopinath, Yi Yuan, Deyou Huang, Liu Miao

**Affiliations:** ^1^Department of Radiology, Liuzhou People's Hospital Affiliated to Guangxi Medical University, Liuzhou, Guangxi 545006, China; ^2^Department of Radiology, Affiliated Hospital of Guilin Medical University, Guilin, Guangxi 541001, China; ^3^Faculty of Chemical Engineering & Technology, Micro System Technology, Centre of Excellence (CoE), and Institute of Nano Electronic Engineering, Universiti Malaysia Perlis (UniMAP), Perlis, Malaysia; ^4^Institute of Life Sciences, Jiangsu University, Zhengjiang, Jiangsu 212013, China; ^5^Department of Radiology, The Affiliated Hospital of Youjiang Medical University for Nationalities, Baise, Guangxi 533000, China; ^6^Department of Cardiology, Liuzhou People's Hospital Affiliated to Guangxi Medical University, Liuzhou, Guangxi 545006, China

## Abstract

**Objective:**

The off-target effects and severe side effects of PPAR*α* and LXR*α* agonists greatly limit their application in atherosclerosis (AS). Therefore, this study intended to use mesoporous silica nanoparticles as carriers to generate MnO nanoparticles in situ with T1WI-MRI in mesoporous pores and simultaneously load PPAR*α* and LXR*α* agonists. Afterward, cRGD-chelated platelet membranes can be used for coating to construct a new nanotheranostic agent.

**Methods:**

cRGD-platelet@MnO/MSN@PPAR*α*/LXR*α* nanoparticles were synthesized by a chemical method. Dynamic light scattering (DLS) was utilized to detect the size distribution and polydispersity index (PDI) of the nanoparticles. The safety of the nanoparticles was detected by CCK8 in vitro and HE staining and kidney function in vivo. Cell apoptosis was detected by flow cytometry detection and TUNEL staining. Oxidative stress responses (ROS, SOD, MDA, and NOX levels) were tested via a DCFH-DA assay and commercial kits. Immunofluorescence and phagocytosis experiments were used to detect the targeting of nanoparticles. Magnetic resonance imaging (MRI) was used to detect the imaging performance of cRGD-platelet@MnO/MSN@PPAR*α*/LXR*α* nanoparticles. Using western blotting, the expression changes in LXR*α* and ABCA1 were identified.

**Results:**

cRGD-platelet@MnO/MSN@PPAR*α*/LXR*α* nanoparticles were successfully established, with a particle size of approximately 150 nm and PDI less than 0.3, and showed high safety both in vitro and in vivo. cRGD-platelet@MnO/MSN@PPAR*α*/LXR*α* nanoparticles showed good targeting properties and better MRI imaging performance in AS. cRGD-platelet@MnO/MSN@PPAR*α*/LXR*α* nanoparticles showed better antioxidative capacities, MRI imaging performance, and diagnostic and therapeutic effects on AS by regulating the expression of LXR*α* and ABCA1.

**Conclusion:**

In the present study, cRGD-platelet@MnO/MSN@PPAR*α*/LXR*α* nanoparticles with high safety and the capacity to target vulnerable plaques of AS were successfully established. They showed better performance on MRI images and treatment effects on AS by promoting cholesterol efflux through the regulation of ABCA1. These findings might address the problems of off-target effects and side effects of nanoparticle-mediated drug delivery, which will enhance the efficiency of AS treatment and provide new ideas for the clinical treatment of AS.

## 1. Introduction

Atherosclerosis (AS) is a chronic disease caused by inflammation in the blood vessel wall, which leads to plaque formation in the endothelial lining in the blood vessel. AS plays a major role in cardiovascular and cerebrovascular-related diseases, which seriously endanger human health [1]. Despite the widespread and successful use of cholesterol-lowering drugs, cardiovascular disease caused by AS is still the leading cause of death worldwide [2]. Kattoor et al. mentioned that reactive oxygen species play a vital role in AS progression [3] and contribute to endothelial injuries [4]. Clarifying the components of AS plaques through auxiliary examinations and assessing the stability of the plaques can provide risk assessment for predicting the occurrence of clinical events. However, the current role of imaging technology is limited to the examination level. The diagnosis of AS still mainly depends on the thickness of the arterial wall and signs of calcification [5]. It is of great significance to identify the components of AS plaques for the targeted treatment of AS.

MRI is a successful imaging technique that is used to diagnose various diseases [6, 7]. With the rapid development of nanoscience and technology, the development of new targeted delivery strategies and new and efficient MRI-T1 contrast agents overcome the cytotoxicity limitations of traditional Gd agents and have pharmacokinetic advantages [8, 9]. This has promoted the successful delivery of the payload to the plaque and realized the diagnosis and treatment of AS [10, 11]. Mesoporous manganese silicate nanoparticles provide a larger surface area for water molecules, and the paramagnetic high-spin metal ions present on the nanoparticle surface have the greatest accessibility to the surrounding water molecules. Therefore, nanoparticles with smaller sizes and larger surface area to volume ratios show a better enhancement effect on T1WI [12]. Therefore, it is necessary to develop a manganese-based MRI-T1 contrast agent to replace the cytotoxic GdIII agent while achieving similar or even better enhancement effects, which has important clinical application value.

The steady state of cholesterol inflow and outflow is of vital importance in the formation of atherosclerosis. With the widespread use of statins, the reduction in cholesterol influx has been clinically successful; however, most cardiovascular-related events still occur due to the plaque load at the beginning of treatment. Therefore, enhancing the cholesterol outflow of atherosclerosis has become the most acceptable treatment to promote AS regression. PPAR and LXR*α* agonists can upregulate the expression of macrophage ABCA1/ABCG1, promote apoA-I-mediated cholesterol efflux, enhance the burial effect of apoptotic cells in the body, and reduce the formation of atherosclerosis in the body [13, 14] and can already be used as oral preparations. However, due to their systemic off-target effects, such as liver steatosis and heart failure, their clinical application is restricted. Therefore, to achieve safe and efficient treatment of AS, it is necessary to develop new noninvasive, targeted diagnosis and therapeutic drug delivery methods for AS.

Platelets are an important part of blood flow and have the ability to maintain blood circulation integrity and help to target vascular injury [15]. It has been demonstrated that modification of nanoparticles with platelet membranes can significantly enhance the targeting of the carrier [16]. Compared with uncoated nanoparticles, platelet membrane-coated nanoparticles can avoid complement activation and the uptake of macrophages, provide nanoparticles with immune escape ability, and can be positioned in deep locations [17]. Neovascularization and macrophages in AS plaques overexpress integrin *α*v*β*3, which can be used to detect the early stages of plaques by targeting the arginine-glycine-aspartate polypeptide loop sequence (cRGD) [18, 19]. Therefore, designing cRGD-modified biointerface platelet membrane-modified nanoparticles for targeted drug delivery within AS plaques is important and difficult and needs to be resolved, in order to provide a new strategy for the clinical treatment of AS. Thus, this study is aimed at constructing mesoporous silica nanoparticles coated with cRGD-platelets and evaluate targeted diagnosis and therapeutic monitoring of AS based on mesoporous silica nanoparticles coated with cRGD-platelets.

## 2. Materials and Methods

### 2.1. cRGD-Platelet@MnO/MSN@PPAR*α*/LXR*α* Nanoparticle Synthesis

Two grams of cetyltrimethylammonium chloride and 0.02 g of triethanolamine were dissolved in 20 mL of water and stirred vigorously, and then the mixed solution was incubated at 80°C for 1 h. Then, 1.5 mL of tetraethyl orthosilicate was added, and stirring was continued for 1 h. The centrifuged product was washed three times with ethanol to eliminate the remaining reactants after centrifugation. Then, CTAC was removed by adding 1 wt% sodium chloride in methanol for 3 h at room temperature. MnOx nanoparticles were introduced into the pores through a redox reaction, and H2 (5%)/Ar (95%) MnO/MSN nanoparticles were obtained under high-temperature reduction. The extracted MnO/MSN was thoroughly washed with ethanol and water and vacuum dried at room temperature (RT). Then, 5 mg MnO/MSNs was dispersed into 6 mL PPAR*α* and LXR*α* agonist PBS solution and stirred at RT for 24 h in the dark, and MnO/MSN/@PPAR*α*/LXR*α* was obtained by centrifugation. The nanoparticles were then added to the platelet membrane and ultrasonicated for 2 min to coat the platelet membrane. The carboxyl-free RGD cyclic peptide molecules were modified to the surface of platelet membrane nanoparticles by the carbodiimide method. Then, the above products and RGD cyclic peptide were mixed in MES buffer and incubated for 30 min. EDC and NHS (0.01 M) were added and placed in a constant temperature shaker at room temperature to react for 24 h. Then, the mixture was centrifuged to remove unreacted RGD cyclic peptide molecules. cRGD-platelet membrane@MnO/MSN@PPAR*α*/LXR*α* nanoparticles were obtained by centrifugation and freeze-dried after washing with DMSO. Dynamic light scattering (DLS) was utilized to detect the size distribution of the nanoparticles.

### 2.2. Particle Size Measurement

The hydrodynamic diameter and polydispersity index (PDI) of MnO/MSN, MnO/MSN@PPAR*α*/LXR*α*, and cRGD-platelet@MnO/MSN@PPAR*α*/LXR*α* were determined using a nanosize analyzer with a dynamic light scattering (DLS) instrument.

### 2.3. Cell Culture and Treatment

THP-1 cells were ordered from the Global Bioresource Center (ATCC, USA), cultured in RPMI 1640 supplemented with 100 U/mL penicillin, fetal bovine serum (10%), and 100 *μ*g/mL streptomycin and placed in a humidified chamber (5% CO_2_ at 37°C). The THP-1 cells were differentiated into macrophages by adding 100 ng/mL PMA for 72 h. The macrophages were transformed into foam cells by incubating for 48 h with 50 *μ*g/mL oxLDL in serum-free RPMI 1640 medium containing 0.3% BSA [20].

### 2.4. CCK-8 Assay

Endothelial cells were seeded in 96-well plates at a density of 1 × 10^4^/well, and then the nanoparticles at different concentrations (0, 5, 10, 20, 100, 1000 *μ*g/mL) were added to the cells and incubated for 24 and 48 h. Culture medium without the nanoparticles was used as a blank control. The viability of endothelial cells was measured using the Cell Counting Kit-8 (Sigma–Aldrich, USA). In brief, a total of 10 *μ*l of CCK-8 solution was added to the cells and incubated for 30 min at 37°C. Absorbance was measured by using a microplate reader (Bio-Rad Laboratories, Inc. Ltd., USA) at 450 nm [21].

### 2.5. Atherosclerosis Model in Rats

Eight-week SPF male Sprague Dawley (SD) rats weighing 200~250 g were purchased from Beijing Vital River Co., Ltd. The AS model in rats was established according to a previous report by feeding with a high-fat diet [22]. The high-fat feed was composed of 20% egg yolk, 5% sugar, 8% lard, and 65% basic feed, fed for 12 weeks, and the AS model was successfully established. Feed was prepared daily, and intake was recorded. After the model was established, the relevant in vivo experiments were started, and the rats with AS were randomly divided into 3 groups, including the control group injected with saline, the cRGD-platelet @MnO/MSN@PPAR*α*/LXR*α* group, and the platelet membrane@MnO/MSN@PPAR*α*/LXR*α* group. The injection was performed by tail vein injection, and all samples were within the safe dose range. ICP–AES quantitative methods were used to evaluate the concentration of diagnostic and therapeutic agents in AS plaques.

### 2.6. Western Blot Analysis

The membranes were incubated in 5% skim milk containing Tween-20 and TRIS-buffered saline for 1 hour. After that, the blocked membranes were placed in a solution containing anti-LXR*α* (1 : 2,000) and anti-ABCA1 (as a loading control, 1 : 1,000) antibodies overnight at 4°C. The next day, the membrane was washed with PBS and then placed in a solution with horseradish peroxidase- (HRP-) conjugated secondary antibody (1 : 5,000) for 1 h. Images were taken by a ChemiDoc MP nucleic acid protein imaging system (Bio-Rad, USA) with enhanced chemiluminescence reagents. Band density was quantified with ImageJ software.

### 2.7. Hematoxylin-Eosin (HE) Staining

Paraffin-embedded tissue samples with nanoparticle treatment were obtained and cut into 4 *μ*m-thick sections. Furthermore, the sections were dipped in hematoxylin staining solution for 3-5 min, and then the slices were rinsed with running water. Subsequently, the slides were dehydrated with 85% and 95% gradient alcohol for 5 min and then stained for 5 min in eosin staining solution. Finally, the cells were washed, images were taken with a microscope (Olympus, Japan) after dehydration, and neutral gum was used to seal the slides.

### 2.8. Immunohistochemical Staining

Paraffin-embedded tissue sections (4 *μ*m thickness) were deparaffinized with xylene and rehydrated using graded alcohols. Hydrogen peroxide with 3% in methanol (50%) was used to block endogenous peroxidase for 10 min at RT. The tissue sections were placed in citrate buffer, heated in a microwave oven for 20 min, and then incubated with primary antibody against PCNA (goat polyclonal, Santa Cruz, sc-9857, 1 : 100 dilution, USA) overnight at 4°C. After that, the slices were washed with PBS and placed in a solution containing biotinylated secondary antibodies, and an avidin-biotinylated peroxidase complex was performed. The color was generated by DAB. Finally, the sections were counterstained with hematoxylin and imaged by a microscope.

### 2.9. Terminal Deoxynucleotidyl Transferase-Mediated d-UTP Nick End Labeling (TUNEL) Assay

Apoptotic cells in tissues were detected by using terminal deoxynucleotidyl transferase-mediated d-UTP nick end labeling (TUNEL). First, sections were immersed in proteinase K (20 min), and deparaffinization and rehydration were conducted. at RT. Then, the sections were placed in TUNEL reaction for 60 minutes at 37°C and washed with PBS thoroughly. Finally, the TUNEL-positive cells labeled with FITC were imaged under fluorescence microscopy (BX-60, Olympus, Japan) with 530 nm emission and 488 nm excitation. Image-Pro Plus 6.0 software was utilized to estimate the number of apoptotic cells [23].

### 2.10. Measurement of Oxidative Stress Response Markers

The levels of ROS in cells and tissues were evaluated using a fluorescent 2′,7′-dichlorofluorescein diacetate (DCFH-DA) assay (Beyotime, China). The cells were seeded on a 96-well black plate at 1 × 10^5^ cells/mL and incubated. The tissues were homogenized and centrifuged. After removing the medium or the supernatant, 10 *μ*M DCFH-DA in PBS was added and maintained for 0.5 h. The fluorescence was measured (ex: 480 nm, em: 530 nm) using a VersaMax microplate reader (MD, USA). The levels of SOD, MDA, and NOX in cells and tissues were measured using commercial detection kits (Beyotime, China) and a VersaMax microplate reader (MD, USA).

### 2.11. Statistical Analysis

The experiments were performed in triplicate and repeated three times. Statistical analyses were performed by utilizing SPSS 21.0 software (SPSS, Inc., USA), and all data were expressed as the means ± standard deviations (SD). Differences between two groups or more than two groups were analyzed by Student's unpaired *t*-test and ANOVA followed by an appropriate post hoc test, respectively. *p* < 0.05 was considered as a significant difference.

## 3. Results

### 3.1. Characteristics of cRGD-Platelet@MnO/MSN@PPAR*α*/LXR*α* Nanoparticles

MnO/MSN, MnO/MSN@PPAR*α*/LXR*α*, and cRGD-platelet@MnO/MSN@PPAR*α*/LXR*α* have particle sizes of ∼130 nm, ∼120 nm, and ∼150 nm, respectively, as determined by DLS (Figure 1(a)). When these nanoparticles were incubated at 4°C for 14 days, there were no significant changes in size or PDI, indicating the intrinsic stability of these nanoparticles (Figure 1(b)). Simultaneously, the zeta potentials of MnO/MSN, MnO/MSN@PPAR*α*/LXR*α*, and cRGD-platelet@MnO/MSN@PPAR*α*/LXR*α* were -41.8 mV, -23.4 mV, and -11.8 mV, respectively. The changing trend of zeta potential suggested that it was reasonable to adopt the synthesis processes (Figure 1(c)). In addition, we found that the drug loading rate was 38.63%, and the encapsulation rate was 98.86% for cRGD-platelet@MnO/MSN@PPAR*α*/LXR*α* (Figures 1(d) and 1(e)). The drug cumulative release reached 80% at 10 h, and cRGD-platelet@MnO/MSN@PPAR*α*/LXR*α* showed the best drug cumulative release curve (Figure 1(f)).

### 3.2. Safety Assessment of cRGD-Platelet@MnO/MSN@PPAR*α*/LXR*α* Nanoparticles

To ensure the safety of the cRGD-platelet@MnO/MSN@PPAR*α*/LXR*α* nanoparticles, the cytotoxicity of the nanoparticles was measured in vitro and in vivo. CCK-8 analysis and flow cytometry analysis indicated that the cell proliferation and apoptosis of foam cell cells were not significantly changed when treated with different concentrations of cRGD-platelet@MnO/MSN@PPAR*α*/LXR*α* nanoparticles (Figures 2(a) and 2(b)). In vivo, routine blood, liver, and kidney function were not affected in all mice treated with different concentrations of cRGD-platelet@MnO/MSN@PPAR*α*/LXR*α* nanoparticles (Figure 2(c)). Meanwhile, no obvious changes were found for the contents of alanine aminotransferase (ALT), aspartate aminotransferase (AST), urea nitrogen (BUN), and creatinine (CREA) in serum injected with different concentrations of cRGD-platelet@MnO/MSN@PPAR*α*/LXR*α* nanoparticles compared with the control group (Figure 2(d)). H&E staining indicated that the tissues presented normal cell morphology, clear boundaries, and orderly tissue structures without inflammation and cell injury treatment with different concentrations of cRGD-platelet@MnO/MSN@PPAR*α*/LXR*α* nanoparticles (Figure 2(e)). In addition, TUNEL and PCNA immunohistochemistry suggested that apoptosis and proliferation were not affected by cRGD-platelet@MnO/MSN@PPAR*α*/LXR*α* nanoparticles at different concentrations (Figures 2(f) and 2(g)). These results indicated that cRGD-platelet@MnO/MSN@PPAR*α*/LXR*α* nanoparticles are safe.

### 3.3. Targeting Performance Evaluation of cRGD-Platelet@MnO/MSN@PPAR*α*/LXR*α* Nanoparticles

The targeting performance of cRGD-platelet@MnO/MSN@PPAR*α*/LXR*α* nanoparticles was detected by laser confocal microscopy at 0.5, 2 h, 4 h, and 8 h in vitro. As shown in Figure 3(a), the fluorescence signals of both cRGD-platelet@MnO/MSN@PPAR*α*/LXR*α* nanoparticles and platelet@MnO/MSN@PPAR*α*/LXR*α* nanoparticles increased with increasing time. However, the fluorescence signal was also significantly increased in the cRGD-platelet@MnO/MSN@PPAR*α*/LXR*α* nanoparticle group compared with the platelet@MnO/MSN@PPAR*α*/LXR*α* group. Furthermore, the T1-MRI signal was enhanced as the concentration of the original nanomaterials increased (Figure 3(b)). The T1-MRI signal was also enhanced in the cRGD-platelet@MnO/MSN@PPAR*α*/LXR*α* nanoparticle group compared with the platelet@MnO/MSN@PPAR*α*/LXR*α* nanoparticle group (Figure 3(b)). In addition, flow cytometry analysis indicated that decreased phagocytosis was observed in the cRGD-platelet@MnO/MSN@PPAR*α*/LXR*α* nanoparticle group compared with the platelet@MnO/MSN@PPAR*α*/LXR*α* nanoparticle group (Figure 3(c)). In addition, we found that the nanoparticles were mainly enriched in the arterial plaque after 4 h (Figure 3(d)). These results demonstrated that cRGD-platelet@MnO/MSN@PPAR*α*/LXR*α* nanoparticles showed good targeting properties in AS.

### 3.4. Diagnostic and Therapeutic Evaluation of cRGD-Platelet@MnO/MSN@PPAR*α*/LXR*α* Nanoparticles

The effect of cRGD-platelet@MnO/MSN@PPAR*α*/LXR*α* nanoparticles on the diagnosis and treatment of AS was assessed. As shown in Figure 4(a), CCK-8 analysis showed that compared with the control group, cell viability was significantly inhibited in both the cRGD-platelet@MnO/MSN@PPAR*α*/LXR*α* and platelet@MnO/MSN@PPAR*α*/LXR*α* nanoparticle groups when the dose was more than 10 *μ*mol/L, and the inhibitory effect was dose-dependent. Flow cytometry and TUNEL assays showed that the apoptosis of cells was significantly elevated when treated with both cRGD-platelet@MnO/MSN@PPAR*α*/LXR*α* and platelet@MnO/MSN@PPAR*α*/LXR*α* nanoparticles compared with the control group (Figures 4(b) and 4(c)). Moreover, the levels of ROS, SOD, MDA, and NOX were evaluated using a DCFH-DA immunofluorescent assay and commercial assay kits. It was reported that both cRGD-platelet@MnO/MSN@PPAR*α*/LXR*α* and platelet@MnO/MSN@PPAR*α*/LXR*α* nanoparticles could reduce cellular oxidative stress responses in contrast to the control group, and cRGD-platelet@MnO/MSN@PPAR*α*/LXR*α* nanoparticles exerted better antioxidative effects than platelet@MnO/MSN@PPAR*α*/LXR*α* nanoparticles (Figures 4(d) and 4(e)). ELISA analysis indicated that the contents of IL-10 and TGF-*β* were significantly decreased when treated with both cRGD-platelet@MnO/MSN@PPAR*α*/LXR*α* and platelet@MnO/MSN@PPAR*α*/LXR*α* nanoparticles compared with the control group (Figure 4(f)). The expression changes of ABCA1 and LXR*α* also confirmed these results (Figure 4(g)). In addition, we found that the diagnostic and therapeutic effects of cRGD-platelet@MnO/MSN@PPAR*α*/LXR*α* nanoparticles against AS were dose-dependent, and cRGD-platelet@MnO/MSN@PPAR*α*/LXR*α* nanoparticles showed better performance and antioxidative capacities than platelet@MnO/MSN@PPAR*α*/LXR*α* nanoparticles (Figures 4(a)–4(g)).

To further confirm the effect of cRGD-platelet@MnO/MSN@PPAR*α*/LXR*α* nanoparticles on the diagnosis and treatment of AS, in vivo experiments were performed with 30 *μ*mol/L cRGD-platelet@MnO/MSN@PPAR*α*/LXR*α* nanoparticles. ICP–AES indicated that the cRGD-platelet@MnO/MSN@PPAR*α*/LXR*α* nanoparticles were significantly enriched in the plaque area and showed better enrichment than platelet@MnO/MSN@PPAR*α*/LXR*α* (Figure 5(a)). HE staining showed that compared with the control group, the area of vascular lesions in the cRGD-platelet@MnO/MSN@PPAR*α*/LXR*α* and platelet@MnO/MSN@PPAR*α*/LXR*α* model groups was significantly decreased (Figure 5(b)). The TUNEL immunofluorescence assay indicated that the intimal injury area and plaque area were significantly decreased when treated with cRGD-platelet@MnO/MSN@PPAR*α*/LXR*α* and platelet@MnO/MSN@PPAR*α*/LXR*α* compared with the control group (Figure 5(c)). Moreover, the levels of ROS, SOD, MDA, and NOX were evaluated using a DCFH-DA assay and commercial assay kits. It was reported that both cRGD-platelet@MnO/MSN@PPAR*α*/LXR*α* and platelet@MnO/MSN@PPAR*α*/LXR*α* nanoparticles could reduce oxidative stress responses in the tissues in contrast to the control group, and cRGD-platelet@MnO/MSN@PPAR*α*/LXR*α* nanoparticles exerted a better antioxidative impact than the platelet@MnO/MSN@PPAR*α*/LXR*α* nanoparticles (Figures 5(d) and 5(e)). The expression of ABCA1 and LXR*α* was significantly elevated in the cRGD-platelet@MnO/MSN@PPAR*α*/LXR*α* and platelet@MnO/MSN@PPAR*α*/LXR*α* groups compared with the control group (Figure 5(f)). These results demonstrated that cRGD-platelet@MnO/MSN@PPAR*α*/LXR*α* nanoparticles showed better diagnostic and therapeutic effects on AS.

## 4. Discussion

Clinical cardiovascular events caused by atherosclerosis (AS) are the leading cause of death worldwide. Efficiently and safely increasing cholesterol efflux and enhancing cell apoptosis have become potential therapeutic methods, but the off-target effects and severe side effects of PPAR*α* and LXR*α* agonists have greatly restricted their clinical applications [2]. To overcome this limitation, predict the occurrence of clinical events, and monitor and evaluate the efficacy of drugs, it is necessary to develop new noninvasive, targeted diagnosis and therapeutic drug delivery methods for AS.

AS is a chronic inflammatory disease. It is an abnormal response of the blood vessel wall to various injuries. It has the characteristics of classic inflammatory degeneration, exudation, and hyperplasia. Vulnerable plaque is characterized by a large lipid pool, a large amount of macrophage aggregation, and thin fibrous caps. They are considered to be markers for identifying vulnerable plaques and evaluation parameters for high risk of future adverse events. The components of AS plaques can be analyzed through auxiliary examinations, and the stability of plaques can be evaluated, in order to provide risk assessment for predicting the occurrence of clinical events [24]. MRI technology has high tissue resolution and can accurately reflect the tissue characteristics of carotid atherosclerotic plaques, including fibrous cap, lipid core, intraplaque hemorrhage, and mural thrombus [25]. Enhanced MRI can show neovascularization, and macrophage infiltration has unique advantages in evaluating vulnerable plaques of the carotid artery [26]. Chen and Schilperoort reviewed macrophage-targeted nanoparticles and nanomedicines designed and applied in the diagnosis and treatment of AS [27]. Liang et al. reported a red blood cell biomimetic nanoparticle for AS treatment that exerted anti-inflammatory, antioxidative, and hypolipidemic effects [28]. In addition, Chyu also studied an apoB-100 peptide-linked nanoparticle to activate immunization against AS progression [29]. In recent years, studies have found that the rate of MRI contrast agent transfer from plasma to the interstitial fluid (Ktrans value) and flowing plasma volume (*vp* value) is significantly and positively correlated with the number of macrophages and new blood vessels [30]. Mesoporous silica has shown great application prospects in biomedicine and other fields due to its ordered mesoporous structure, large specific surface area, good biocompatibility, and easy surface modification, such as in MRI contrast agents, bioimaging, and nanodrug delivery systems [31, 32]. For example, Menard et al. designed hybrid protein-coated magnetic core-mesoporous silica shell nanocomposites that could be used for MRI and drug release in a 3D tumor cell model [33]. Chen et al. established an RGD-modified and pyroptosis-engineered theranostic agent (PETA) consisting of Fe3O4-embedded magnetic mesoporous silica nanoparticle (MMSN) vehicles and chlorin e6 (Ce6) photosensitizers to strengthen ROS levels to trigger pyroptosis by a Ce6-mediated photodynamic process [34]. Yang et al. developed a urine microenvironment-responsive 3D-printed hydrogel patch for realizing scarless memory repair, wherein laser-excited reactive oxygen species production and mechanical strength elevation were achieved using chemically crosslinked silicon quantum dots [35]. Kong et al. used a Nb2C/Au nanocomposite to demonstrate a microbiome metabolism-engineered phototherapy strategy in the regulation of bacteria [36]. A biomimetic Sim@PMPB theranostic agent designed by Zhang et al. successfully stabilized atherosclerotic plaques, alleviated atherosclerosis, and localized and amplified atherosclerosis, enabling monitoring of H_2_O_2_-related atherosclerotic evolution after treatment [37]. Li et al. indicated that mesoporous manganese silicate-coated silica nanoparticles could be used as multistimuli-responsive T1-MRI contrast agents and drug delivery carriers [38]. Chen et al. found that mesoporous manganese silicate nanoparticles show better enhancement effects on T1WI due to their smaller size and the higher surface-area-to-volume ratio [12]. Therefore, it is necessary to develop a manganese-based MRI-T1 contrast agent to replace the cytotoxic GdIII agent while achieving similar or even better enhancement effects, which is extremely challenging and has clinical application value. In this study, we developed a cRGD-platelet@MnO/MSN@PPAR*α*/LXR*α* nanoparticle that showed high safety both in vitro and in vivo. Further analysis revealed that cRGD-platelet@MnO/MSN@PPAR*α*/LXR*α* nanoparticles showed better MRI imaging performance in AS.

In fact, most of the nanoformulations are not sufficiently targeted in vivo and are easily cleared by mononuclear macrophages. Platelets are an important part of blood flow and have the ability to target vascular injury sites and maintain the integrity of blood circulation [39, 40]. Bai et al. wrapped Fe_3_O_4_ magnetic nanoparticles with platelet membranes for tumor MRI and photothermal therapy. It was found that platelet membrane-modified magnetic nanoparticles had a longer blood circulation time and better tumor-targeting properties, significantly improved the effects of MRI and photothermal therapy, and had good in vivo safety [41]. Zha et al. used platelet membranes to prepare nanomedicine with photodynamic/photothermal synergistic therapy. Nanomedicine can circulate in the body for a long time, can effectively target tumor cells, and is beneficial to the penetration of deep tumor tissues [42]. These results suggested that the platelet membrane-coated nanoparticles can avoid complement activation and the uptake of macrophages, provide the nanoparticles with immune escape ability, and can be located in deep locations. In addition, integrin *α*v*β*3 is an important marker of angiogenesis, and cRGD is currently known to specifically bind to integrin *α*v*β*3. Increasing numbers of RGD probes have been applied by targeting *α*v*β*3. Studies have found that new blood vessels in AS plaques and macrophages overexpress integrin *α*v*β*3, which provides the basis for the application of cRGD in targeting vulnerable plaques by targeting *α*v*β*3 [18, 19]. The current investigation demonstrated that cRGD-platelet@MnO/MSN@PPAR*α*/LXR*α* nanoparticles showed better performance than platelet@MnO/MSN@PPAR*α*/LXR*α* nanoparticles, suggesting that cRGD-platelet@MnO/MSN@PPAR*α*/LXR*α* nanoparticles had better diagnostic and therapeutic effects on AS.

In atherosclerotic plaques, cholesterol efflux is reduced, and the continuous accumulation of free cholesterol in foam cells leads to endoplasmic reticulum stress, inflammatory reactions, and finally foam cell apoptosis. If the apoptotic bodies cannot be effectively cleared by the burial effect, necrosis will occur, leading to the progression of atherosclerosis [43]. Therefore, the steady state of cholesterol inflow and outflow is of vital importance in the formation of atherosclerosis. The PPAR-LXR*α*-ABCA1/ABCG1 pathway of macrophages plays an important role in regulating cholesterol efflux. In addition to regulating cholesterol homeostasis, PPAR*α* and LXR*α* can also exhibit anti-inflammatory functions by preventing the release of inflammatory cytokines [44, 45]. In addition, we also found that the application of platelet@MnO/MSN@PPAR*α*/LXR*α* nanoparticles and cRGD-platelet@MnO/MSN@PPAR*α*/LXR*α* nanoparticles had antioxidative effects, and that cRGD-platelet@MnO/MSN@PPAR*α*/LXR*α* nanoparticles had stronger antioxidative abilities than platelet@MnO/MSN@PPAR*α*/LXR*α* nanoparticles. PPAR*α* is a ligand-activated transcription factor, and its target genes control oxidative stress in rats. The activation of PPAR*α* mediates oxidative stress responses [46, 47].

In addition, activated LXR*α* elevates the phagocytosis of apoptotic cells by inducing the expression of the cell surface receptor Mer tyrosine kinase (MerTK) [48]. The expression level of LXR*α* was also associated with cellular inflammation and oxidative stress responses [49]. All these results indicate that the activation of PPAR*α* and LXR*α* improves the prognosis of AS patients. Studies have found that the combination of PPAR*α* and LXR*α* agonists can reduce the adverse effects of a single use of agonists. It is speculated that PPAR*α* agonists may change the plasma TG concentration. Therefore, it is speculated that the combination of PPAR*α* agonists and LXR*α* agonists may reduce the risk of AS, which is particularly effective and is considered to be a promising treatment strategy [50, 51]. However, the mechanism of this strategy for treating AS has not yet been elucidated. Additionally, due to their systemic off-target effects, such as liver steatosis and heart failure, their clinical applications are limited. The current study demonstrated that the cholesterol contents were significantly decreased when treated with cRGD-platelet@MnO/MSN@PPAR*α*/LXR*α* nanoparticles compared with the control group. The expression of ABCA1 and LXR*α* was significantly elevated when treated with cRGD-platelet@MnO/MSN@PPAR*α*/LXR*α*. These results suggested that cRGD-platelet@MnO/MSN@PPAR*α*/LXR*α* nanoparticles alleviated AS development by promoting cholesterol effluence by regulating the expression of ABCA1 and LXR*α*. Molecular imaging of atherosclerosis was performed with nanoparticle-based fluorinated MRI contrast agents.

Finally, this study has several limitations; for example, the safety and efficacy of cRGD-platelet@MnO/MSN@PPAR*α*/LXR*α* nanoparticles should be monitored long-term. Next, different species of model animals should be used to test the effects of this nanoparticle. Finally, the underlying mechanisms and molecular pathways involved in the therapeutic effects of this nanoparticle should also be investigated.

## 5. Conclusion

In summary, we successfully established cRGD-platelet@MnO/MSN@PPAR*α*/LXR*α* nanoparticles with high safety and targeting of vulnerable plaques of AS. Further analysis showed that cRGD-platelet@MnO/MSN@PPAR*α*/LXR*α* nanoparticles had better performance on MRI imaging and treatment effects on AS by promoting cholesterol efflux through the regulation of ABCA1.

These findings suggested that the risk prediction, treatment, monitoring, and evaluation of AS might be realized by mesoporous silica nanoparticles coated with cRGD-platelets, which can provide a basis for the clinical diagnosis of AS and has broad application prospects. Our findings provide a reference for solving the off-target and side effects of nanoparticle-mediated drug delivery, improving the efficiency of AS treatment, and providing new ideas for the clinical treatment of AS.

## Figures and Tables

**Figure 1:** Characteristics of cRGD-platelet@MnO/MSN@PPAR*α*/LXR*α* nanoparticles. (a) DLS diameters of MnO/MSN, MnO/MSN@PPAR*α*/LXR*α*, and cRGD-platelet@MnO/MSN@PPAR*α*/LXR*α*. (b) The variations in particle size and PDI of cRGD-platelet@MnO/MSN@PPAR*α*/LXR*α* at 4°C for 14 days. (c) The zeta potential of cRGD-platelet@MnO/MSN@PPAR*α*/LXR*α*. (d, e) Drug loading rate and the encapsulation rates for cRGD-platelet@MnO/MSN@PPAR*α*/LXR*α*, respectively. (f) Drug cumulative release of cRGD-platelet@MnO/MSN@PPAR*α*/LXR*α*; *n* = 1 for (a)–(c) and (f); *n* = 3 for (d) and (e).

**Figure 2:** Safety assessment of cRGD-platelet@MnO/MSN@PPAR*α*/LXR*α* nanoparticles. (a) CCK-8 was used to detect the proliferation of THP-1 cells and foam cells treated with different nanoparticles. (b) Flow cytometry assay was used to detect the apoptosis of foam cells treated with different nanoparticles. (c) The routine blood, liver, and kidney function were detected by ELISA after treatment with different concentrations of nanoparticles. (d) The contents of ALT, AST, BUN, and CREA in serum injected with different concentrations of nanoparticles. (e) H&E staining was utilized to detect the status of the tissue in different organs treated with different concentrations of nanoparticles. (f, g) TUNEL and PCNA immunohistochemistry were used to detect the changes in apoptosis and proliferation after treatment with nanoparticles at different concentrations. Data are shown as the mean ± SD. *n* = 1 for (b) and (e)–(g); *n* = 3 for (a), (c), and (d).

**Figure 3:** Targeting performance evaluation of cRGD-platelet@MnO/MSN@PPAR*α*/LXR*α* nanoparticles. (a) The fluorescence signal of nanoparticles detected by laser confocal microscopy at 0.5, 2 h, 4 h, and 8 h in vitro. (b) The T1-MRI signal was enhanced as the concentration of the original nanomaterials increased. (c) Flow cytometry analysis was utilized to detect the phagocytosis affected by nanoparticles. (d) ICP–AES was utilized to detect the enrichment of cRGD-platelet@MnO/MSN@PPAR*α*/LXR*α* nanoparticles in the arterial plaque. Data are shown as the mean ± SD, ^∗∗^*p* < 0.01 vs. platelet@MnO/MSN@PPAR*α*/LXR*α*. *n* = 1 for (a) and (c); *n* = 3 for (b) and (d).

**Figure 4:** Diagnostic and therapeutic evaluation of cRGD-platelet@MnO/MSN@PPAR*α*/LXR*α* nanoparticles in vitro. (a) Cell viability was detected by CCK-8 after treatment with different nanoparticles. (b, c) Flow cytometry and TUNEL assays were utilized to determine the apoptosis of cells treated with cRGD-platelet@MnO/MSN@PPAR*α*/LXR*α*. (d) The level of ROS was detected by DCFH-DA immunofluorescent assay. (e) The levels of SOD, MDA, and NOX were evaluated using commercial assay kits. (f) ELISA analysis was used to detect the contents of IL-10 and TGF-*β* after treatment with cRGD-platelet@MnO/MSN@PPAR*α*/LXR*α*. (g) The expression changes of ABCA1 and LXR*α* were determined by western blot after treatment with the cRGD-platelet@MnO/MSN@PPAR*α*/LXR*α*. Data are shown as the mean ± SD, ^∗∗^*p* < 0.01 vs. control. *n* = 1 for (c) and (d); *n* = 3 for (a), (b), (e), (f), and (g).

**Figure 5:** Diagnostic and therapeutic evaluation of cRGD-platelet@MnO/MSN@PPAR*α*/LXR*α* nanoparticles in vivo. (a) ICP–AES was utilized to determine the enrichment of the cRGD-platelet@MnO/MSN@PPAR*α*/LXR*α* nanoparticles in the plaque area. (b) HE staining was used to detect the area of vascular lesions affected by cRGD-platelet@MnO/MSN@PPAR*α*/LXR*α*. (c) TUNEL immunofluorescence assay was used to detect the intimal injury area and plaque area when treated with cRGD-platelet@MnO/MSN@PPAR*α*/LXR*α*. (d) The level of ROS was detected by DCFH-DA assay. (e) The levels of SOD, MDA, and NOX were evaluated using commercial assay kits. (f) The expression of ABCA1 and LXR*α* was detected by western blot after treatment with the cRGD-platelet@MnO/MSN@PPAR*α*/LXR*α*. Data were displayed as the mean ± SD, ^∗∗^*p* < 0.01 vs. control. *n* = 1 for (b) and (c); *n* = 3 for (a), (d), (e), and (f).

## Data Availability

The datasets used and analyzed in the current study would be available from the corresponding author upon request.

## References

[1] Milutinovic A., Suput D., Zorc-Pleskovic R. (2020). Pathogenesis of atherosclerosis in the tunica intima, media, and adventitia of coronary arteries: an updated review. *Bosnian Journal of Basic Medical Sciences*.

[2] Frostegard J. (2013). Immunity, atherosclerosis and cardiovascular disease. *BMC medicine*.

[3] Kattoor A. J., Pothineni N. V. K., Palagiri D., Mehta J. L. (2017). Oxidative stress in atherosclerosis. *Current Atherosclerosis Reports*.

[4] Malekmohammad K., Sewell R. D., Rafieian-Kopaei M. (2019). Antioxidants and atherosclerosis: Mechanistic aspects. *Biomolecules*.

[5] Andreini D., Magnoni M., Conte E. (2020). Coronary plaque features on CTA can identify patients at increased risk of cardiovascular events. *JACC: Cardiovascular Imaging*.

[6] Kocaoglu M., Kline-Fath B. M., Calvo-Garcia M. A., Zhang B., Nagaraj U. D. (2020). Magnetic resonance imaging of the fetal brain in monochorionic diamniotic twin gestation: correlation of cerebral injury with ultrasound staging and survival outcomes. *Pediatric Radiology*.

[7] Shukla G., Alexander G. S., Bakas S. (2017). Advanced magnetic resonance imaging in glioblastoma: a review. *Chinese Clinical Oncology*.

[8] Yousaf T., Dervenoulas G., Politis M. (2018). Advances in MRI methodology. *International Review of Neurobiology*.

[9] Geethanath S., Vaughan J. T. (2019). Accessible magnetic resonance imaging: a review. *Journal of Magnetic Resonance Imaging*.

[10] Phinikaridou A., Andia M. E., Lacerda S., Lorrio S., Makowski M., Botnar R. (2013). Molecular MRI of atherosclerosis. *Molecules*.

[11] Zhou L., Yan Y., Du H., Ni X., Wang G., Wang Q. (2020). Plaque features and vascular geometry in basilar artery atherosclerosis. *Medicine (Baltimore)*.

[12] Chen Y., Chen H., Shi J. (2013). In vivo bio-safety evaluations and diagnostic/therapeutic applications of chemically designed mesoporous silica nanoparticles. *Advanced Materials*.

[13] Schumacher T., Benndorf R. A. (2017). ABC transport proteins in cardiovascular disease-a brief summary. *Molecules*.

[14] Zeng Y., Peng Y., Tang K. (2018). Dihydromyricetin ameliorates foam cell formation via LXR*α*- ABCA1/ABCG1-dependent cholesterol efflux in macrophages. *Biomedicine & Pharmacotherapy*.

[15] Thon J. N., Italiano J. E. (2012). Platelets: production, morphology and ultrastructure. *Handbook of Experimental Pharmacology*.

[16] Wang H., Liu Y., He R. (2020). Cell membrane biomimetic nanoparticles for inflammation and cancer targeting in drug delivery. *Biomaterials Science*.

[17] Choi B., Park W., Park S. B., Rhim W. K., Han D. K. (2020). Recent trends in cell membrane-cloaked nanoparticles for therapeutic applications. *Methods*.

[18] Kim M., Sahu A., Kim G. B. (2018). Comparison of *in vivo* targeting ability between cRGD and collagen-targeting peptide conjugated nano-carriers for atherosclerosis. *Journal of Controlled Release*.

[19] Razavian M., Marfatia R., Mongue-Din H. (2011). Integrin-targeted imaging of inflammation in vascular remodeling. *Arteriosclerosis, Thrombosis, and Vascular Biology*.

[20] Lomovskaya Y. V., Kobyakova M. I., Senotov A. S. (2022). Macrophage-like THP-1 Cells Derived from High-Density Cell Culture Are Resistant to TRAIL-Induced Cell Death via Down-Regulation of Death-Receptors DR4 and DR5. *Biomolecules*.

[21] Liu L., Guo H., Song A. (2020). Progranulin inhibits LPS-induced macrophage M1 polarization via NF-кB and MAPK pathways. *BMC Immunology*.

[22] Subramani C., Rajakannu A., Gaidhani S., Raju I., Kartar Singh D. V. (2020). Glutathione-redox status on hydro alcoholic root bark extract of *Premna integrifolia* Linn in high fat diet induced atherosclerosis model. *Journal of Ayurveda and integrative medicine*.

[23] Xie C., Zhou X., Liang C. (2021). Apatinib triggers autophagic and apoptotic cell death via VEGFR2/STAT3/PD-L1 and ROS/Nrf2/p62 signaling in lung cancer. *Journal of Experimental & Clinical Cancer Research*.

[24] Ruiz-León A. M., Lapuente M., Estruch R., Casas R. (2019). Clinical advances in immunonutrition and atherosclerosis: a review. *Frontiers in immunology*.

[25] Harisinghani M. G., O’Shea A., Weissleder R. (2019). Advances in clinical MRI technology. *Science Translational Medicine*.

[26] Palekar R. U., Jallouk A. P., Lanza G. M., Pan H., Wickline S. A. (2015). Molecular imaging of atherosclerosis with nanoparticle-based fluorinated MRI contrast agents. *Nanomedicine (London, England)*.

[27] Chen W., Schilperoort M., Cao Y., Shi J., Tabas I., Tao W. (2022). Macrophage-Targeted Nanomedicine for the Diagnosis and Treatment of Atherosclerosis. *Nature reviews Cardiology*.

[28] Liang X., Li H., Zhang A. (2022). Red blood cell biomimetic nanoparticle with anti-inflammatory, anti-oxidative and hypolipidemia effect ameliorated atherosclerosis therapy. *Nanomedicine*.

[29] Chyu K. Y., Zhao X., Zhou J. (2022). Immunization using ApoB-100 peptide-linked nanoparticles reduces atherosclerosis. *JCI insight*.

[30] Wang J., Chen H., Sun J. (2017). Dynamic contrast-enhanced MR imaging of carotid *vasa vasorum* in relation to coronary and cerebrovascular events. *Atherosclerosis*.

[31] Wang Y., Zhao Q., Han N. (2015). Mesoporous silica nanoparticles in drug delivery and biomedical applications. *Nanomedicine*.

[32] McCarthy C. A., Ahern R. J., Dontireddy R., Ryan K. B., Crean A. M. (2016). Mesoporous silica formulation strategies for drug dissolution enhancement: a review. *Expert Opinion on Drug Delivery*.

[33] Ménard M., Meyer F., Affolter-Zbaraszczuk C. (2019). Design of hybrid protein-coated magnetic core-mesoporous silica shell nanocomposites for MRI and drug release assessed in a 3D tumor cell model. *Nanotechnology*.

[34] Chen M., Liao H., Bu Z. (2022). Pyroptosis activation by photodynamic-boosted nanocatalytic medicine favors malignancy recession. *Chemical Engineering Journal*.

[35] Yang M., Zhang Y., Fang C. (2022). Urine-microenvironment-initiated composite hydrogel patch reconfiguration propels scarless memory repair and reinvigoration of the urethra. *Advanced Materials*.

[36] Kong F., Fang C., Zhang Y. (2022). Abundance and metabolism disruptions of intratumoral microbiota by chemical and physical actions unfreeze tumor treatment resistance. *Advanced Science*.

[37] Zhang Y., Yin Y., Zhang W. (2021). Reactive oxygen species scavenging and inflammation mitigation enabled by biomimetic prussian blue analogues boycott atherosclerosis. *Journal of nanobiotechnology*.

[38] Li X., Zhao W., Liu X. (2016). Mesoporous manganese silicate coated silica nanoparticles as multi-stimuli- responsive T_1_-MRI contrast agents and drug delivery carriers. *Acta Biomaterialia*.

[39] Ho-Tin-Noe B., Boulaftali Y., Camerer E. (2018). Platelets and vascular integrity: how platelets prevent bleeding in inflammation. *Blood, The Journal of the American Society of Hematology*.

[40] Liu X., Zhang F., Wang Q. (2014). Platelet-inspired multiscaled cytophilic interfaces with high specificity and efficiency toward point-of-care cancer diagnosis. *Small*.

[41] Bai Y., Zhang Y., Zhang J. (2010). Repeated administrations of carbon nanotubes in male mice cause reversible testis damage without affecting fertility. *Nature Nanotechnology*.

[42] Zha Z., Wang J., Zhang S. (2014). Engineering of perfluorooctylbromide polypyrrole nano-/microcapsules for simultaneous contrast enhanced ultrasound imaging and photothermal treatment of cancer. *Biomaterials*.

[43] Koelwyn G. J., Corr E. M., Erbay E., Moore K. J. (2018). Regulation of macrophage immunometabolism in atherosclerosis. *Nature Immunology*.

[44] Bensinger S. J., Tontonoz P. (2008). Integration of metabolism and inflammation by lipid-activated nuclear receptors. *Nature*.

[45] Ruan X. Z., Moorhead J. F., Fernando R., Wheeler D. C., Powis S. H., Varghese Z. (2003). PPAR agonists protect mesangial cells from interleukin 1beta-induced intracellular lipid accumulation by activating the ABCA1 cholesterol efflux pathway. *Journal of the American Society of Nephrology*.

[46] Pawlak M., Lefebvre P., Staels B. (2015). Molecular mechanism of PPAR*α* action and its impact on lipid metabolism, inflammation and fibrosis in non-alcoholic fatty liver disease. *Journal of Hepatology*.

[47] Zhang Y., Cui Y., Wang X. L. (2015). PPAR*α*/*γ* agonists and antagonists differently affect hepatic lipid metabolism, oxidative stress and inflammatory cytokine production in steatohepatitic rats. *Cytokine*.

[48] Doran A. C., Ozcan L., Cai B. (2017). CAMKII*γ* suppresses an efferocytosis pathway in macrophages and promotes atherosclerotic plaque necrosis. *The Journal of Clinical Investigation*.

[49] Jia Q., Cao H., Shen D. (2019). Quercetin protects against atherosclerosis by regulating the expression of PCSK9, CD36, PPAR*γ*, LXR*α* and ABCA1. *International Journal of Molecular Medicine*.

[50] Beyer T. P., Schmidt R. J., Foxworthy P. (2004). Coadministration of a liver X receptor agonist and a peroxisome proliferator activator receptor-alpha agonist in mice: effects of nuclear receptor interplay on high-density lipoprotein and triglyceride metabolism in vivo. *The Journal of Pharmacology and Experimental Therapeutics*.

[51] Marchi C., Adorni M. P., Caffarra P. (2019). ABCA1- and ABCG1-mediated cholesterol efflux capacity of cerebrospinal fluid is impaired in Alzheimer’s disease. *Journal of Lipid Research*.

